RETRACTED

# Comprehensive Analysis of Mango (*Mangifera indica* L.) Seed: Phytochemical Profile, Bioactivity, and Nutraceutical Potential

**DOI:** 10.1002/fsn3.70390

**Published:** 2025-06-16

**Authors:** Shafa Iman, Mamoon ur Rasheed, Hamdy A. Zahran, Haroon Rashid, Mehak Fatima, Zonish Saleem, Yasmeen Bano, Sanobar Gull, Raheeba Akbar, Ayesha Khan, Isam A. Mohamed Ahmed, Eliasse Zongo, Muhammad Abdul Rahim, Roberto Castro‐Muñoz

**Affiliations:** ^1^ Department of Pharmacology, Faculty of Pharmaceutical Sciences Government College University Faisalabad Pakistan; ^2^ Department of Chemistry Government College University Faisalabad Pakistan; ^3^ Fats and Oils Department, Food Industries and Nutrition Research Institute National Research Centre Cairo Egypt; ^4^ Department of Physiology, Faculty of Veterinary and Animal Sciences The Islamia University of Bahawalpur Bahawalpur Pakistan; ^5^ National Institute of Food Science and Technology University of Agriculture Faisalabad Pakistan; ^6^ Department of Chemistry University of Agriculture Faisalabad (UAF) Faisalabad Pakistan; ^7^ Department of Food Science and Nutrition, College of Food and Agricultural Sciences King Saud University Riyadh Saudi Arabia; ^8^ Laboratoire de Recherche et D'enseignement en Santé et Biotechnologies Animales Université Nazi BONI Bobo Dioulasso Burkina Faso; ^9^ Department of Food Science & Nutrition, Faculty of Medicine and Allied Health Sciences Times University Multan Pakistan; ^10^ Department of Sanitary Engineering, Faculty of Civil and Environmental Engineering Gdańsk University of Technology Gdansk Poland

**Keywords:** FTIR, GC–MS, mango ( *Mangifera indica* L.) seeds, nutritional analysis

## Abstract

Mango ( *Mangifera indica* L.) seeds, typically discarded as agro‐industrial waste, are rich in bioactive compounds with significant nutraceutical potential. This study comprehensively evaluated the phytochemical composition, cytotoxicity, antioxidant activity, nutritional profile, and safety of mango seed extract (MSE). Nutritional analysis revealed notable contents of crude protein (8.5% ± 0.01%), crude oil (13.5% ± 0.06%), carbohydrates (35% ± 0.01%), and energy (405 kJ/100 g) while mineral content indicates the presence of macrominerals in the following order: K > Mg > P > Ca > Na. GC–MS identified key bioactive compounds, including thiazole, silicic acid, and arsenic acid. MSE exhibited strong antioxidant activity, with 95.86% ± 2.31% DPPH and 89.36% ± 5.25% nitric oxide radical scavenging. Cytotoxicity assays against HepG2 liver cancer cells demonstrated dose‐dependent inhibition, with an IC_50_ of 140 μg/mL. Nutritional analysis showed essential amino acids (lysine, leucine, valine) and vitamins A, C, E, and K. Molecular dynamic simulations (MDS) confirmed thiazole's binding affinity to estrogen‐β and progesterone receptors. Subacute oral toxicity tests indicated MSE's safety and beneficial effects on lipid profiles, significantly reducing cholesterol, LDL, triglycerides, and VLDL, while increasing HDL and RBC counts. Histopathology confirmed no organ damage. These results establish MSE as a safe, sustainable source of bioactive compounds with promising applications in nutraceuticals, antioxidants, and functional food industries, offering an eco‐friendly approach to mango seed waste valorization.

RETRACTED

## Graphical abstract

The cytotoxic effects of the MI plant were studied through MTT assay, which revealed its potential to inhibit growth against HepG2 cell lines. FTIR analysis confirms the various functional groups. Various bioactive constituents were identified from the LC–MS investigation of aqueous methanol extracts of MSE, exhibiting the existence of various phytochemical activities. MI workflow provides a comprehensive paradigm for exploring ligand‐protein interactions based on classical molecular dynamics, including the simulations and their analysis. The results from the in vitro and in vivo analysis showed that extracts of MI possess antioxidant, hepatoprotective, and nephroprotective potential and serve as potential therapeutic agents in combating diabetes mellitus (DM). Further studies should be designed to explore the mechanistic approaches of the bioactive constituents in the MI plant.

## 1 Introduction

The increasing global production of mango has led to a significant rise in the generation of agro‐industrial waste, particularly mango seeds, which account for 20%–60% of the fruit's weight. Annually, approximately 14–25 million tons of mango by‐products are discarded, contributing to environmental pollution and waste management challenges (Torres‐León et al. 2021; Gianazza et al. 2019). Despite their disposal as waste, mango seeds are rich in bioactive compounds with potential health benefits, including antioxidant, anti‐inflammatory, and immunomodulatory properties (Torres‐León et al. 2021; Castro‐Muñoz et al. 2024).

Toxic compounds are produced when human lipoproteins and lipids undergo autoxidation and oxidative stress. Nowadays, oxidative stress is considered the leading cause of various ailments such as cancer, diseases of the heart and nervous system, diabetes, and aging (Gianazza et al. 2019; Liu et al. 2025; Castro‐Muñoz et al. 2022). In underdeveloped nations, herbal remedies have been the mainstay of medical care. The plants naturally contain the antioxidant potential that could be used in the prevention or treatment of numerous ailments (Hernández‐Pinto et al. 2024). Therefore, this potential reinforces the initiative to investigate natural agents as an alternative to synthetic medications. The usage of synthetic chemicals is expensive and confined due to complexity and untoward effects on human health (Gaston et al. 2020; Ferreyra‐Suarez et al. 2024). Mango, scientifically known as *Mangifera indica* , is a member of the Anacardiaceae family and is indigenous to tropical regions. Renowned for its juicy and delicious flavor, the mango is highly appreciated worldwide. The fruit varies significantly in size, shape, sweetness, and color, with cultivars exhibiting hues ranging from green to yellow, red, and orange. Its rich nutritional profile makes it a popular choice among consumers, contributing to its status as one of the most widely cultivated fruits globally.

RETRACTED

It is a tropical fruit and is significantly enjoyed for its juiciness and delightful flavor in most of the states of the world (Garza‐Cadena et al. 2023). While processing ripped fruit, the seeds are discarded, which may significantly raise ecological contamination (Yadav and Paudel 2022; Sagar et al. 2018). From an ecological viewpoint, it is essential to recycle plant waste formed by the food industry (Laskar et al. 2020). The health‐promoting properties of mango seeds and their bioactive components have been covered in several reviews (Lebaka et al. 2021). It has been reported that mango seeds have an excellent content of minerals: iron, sodium, calcium, magnesium, potassium, phosphorus, and vitamins (Rai et al. 2020). In underdeveloped nations, mango seeds are used as a substitute for flour and in animal feed to deal with the issue of food scarcity (Beriso and Tesfaye 2024). The phytochemical evaluation revealed the presence of phenols, Mangiferin, flavonoids, glucosyl xanthone, gallic acid, coumarin, caffeic acid, vanillin, Mangiferin, ferulic acid, and cinnamic acid in mango seeds.

Various pharmacological evaluations by other researchers showed that mango seeds contain antioxidant, anti‐tyrosinase, anti‐inflammatory, anticancer, hepatoprotective, and immune‐modulatory actions (Rai et al. 2020). It has been reported in a previous study that mango possesses antidiabetic potential, as shown by the decrease in the postprandial blood glucose level. Furthermore, it increases glucose tolerance, lipid profile, improves body weight, and decreases the damage to beta cells (Saleem et al. 2019). Comprehensive studies evaluating its cytotoxic potential specifically against HepG2 cell lines and detailed subacute toxicity profiles remain limited. This study aims to explore the nutritional attributes and phytochemical profile of MSE, highlighting their value as a sustainable resource that can mitigate ecological issues while promoting health (Ganogpichayagrai et al. 2017). By investigating the cytotoxic and nutraceutical features of mango seed extracts, this research seeks to uncover their potential applications in the food and pharmaceutical industries, thereby addressing both waste reduction and health enhancement.

RETRACTED

## 2 Materials and Methods

Various varieties of mango seed extracts (MSE) were sourced from local markets in Faisalabad (Coordinates: 31°25′0″ N 73°5′28″ E) between May and August 2022. After removing the hairy coating, the seeds were collected, dried at room temperature, and ground into a fine flour. The seeds were identified and authenticated by Dr. Mansoor Hameed, a taxonomist from the Department of Botany at the University of Agriculture Faisalabad (UAF) and were deposited in the herbarium under voucher number 79‐1‐2019.

### 2.1 Extract Preparation

A total of 500 g of dried MSE was immersed in a solvent mixture of aqueous methanol (20:80) for 72 h, with intermittent stirring to enhance extraction. Following this period, the mixture was filtered using Whatman filter paper No. 1 to separate the solid residues from the liquid extract. The resulting extract was then concentrated under reduced pressure using a rotary evaporator at a temperature of 40°C.

### 2.2 Nutritional Composition of MSE

A chemical examination of MSE was conducted to determine its ash, crude protein, fiber, fat, and mineral content (including calcium, magnesium, potassium, sodium, and phosphorus), following the standard methods outlined by the Association of Official Analytical Chemists (Sambucetti and Zuleta 1996). Additionally, carbohydrate and energy contents were calculated. Each parameter was calculated in triplicate to ensure accuracy, and average values were recorded for each measurement (Lebaka et al. 2021).

### 2.3 Evaluation of Amino Acid

For the evaluation of amino acid content in the given sample, the isolated protein from the MSE was formed by the addition of 6 N HCl into a pestle and mortar. After filtering it (250 mL), the sample protein was hydrolyzed by retaining the flask in a heating mantle for 30 min at 100°C. To evaporate HCl, the resultant mixture was placed in a water bath. Again, filter it with 0.1 N HCl (stock solution). Subsequently, filter the stock solution with a 0.45 μm syringe filter. Finally, stock and standard solutions were run through the amino acid analyzer (Ojha et al. 2019).

### 2.4 Determination of Vitamins

The levels of vitamins C, A, E, and K in mango seed extract (MSE) were determined following the official method (Sambucetti and Zuleta 1996). For sample preparation, 10 g of MSE was extracted with 50 mL of ethanol, allowed to stand for 30 min, and filtered through Whatman filter paper. The filtered extract underwent saponification by adding 25 mL of 0.5 N sodium hydroxide (NaOH) and heating gently for 30 min while stirring. After cooling, the mixture was neutralized with hydrochloric acid (HCl) to achieve a neutral pH. A liquid–liquid extraction was performed by adding hexane to the neutralized solution, shaking vigorously, and separating the upper hexane layer containing fat‐soluble vitamins A and E. The hexane was evaporated using a rotary evaporator at 40°C, and the residue was dissolved in methanol for analysis. Vitamins A and E were quantified using high‐performance liquid chromatography (HPLC) equipped with a UV detector for retinol (vitamin A) at 328 nm and a fluorescence detector for alpha‐tocopherol (vitamin E) with excitation at 290 nm and emission at 330 nm. Vitamin C was analyzed by dissolving an aliquot of MSE in distilled water and measuring absorbance using a spectrophotometer. For vitamin K, saponified extracts were processed with acetone and analyzed via HPLC with fluorescence detection (Sambucetti and Zuleta 1996). All analyses were performed in triplicate, and concentrations were calculated using standard calibration curves. Results were reported as mg of each vitamin per gram of MSE, ensuring accuracy and reliability in quantifying the nutritional composition of the extract (Sarkar et al. 2022).

RETRACTED

### 2.5 Phytochemical Assay

MSE was assessed for the existence of different phytochemicals present in it (Fitmawati et al. 2020).

### 2.6 Test for Alkaloid

To assess the presence of alkaloids within the mango seed extract (MSE), a series of established qualitative tests was employed. For the alkaloid determination, 2 mL of the MSE extract was initially mixed with 2 N hydrochloric acid (HCl). The resulting mixture was then filtered to remove any particulate matter. Subsequently, an equal volume (2 mL) of Dragendorff's reagent was added to the filtrate. The observation of an orange precipitate indicated the presence of alkaloids within the extract. The formation of this precipitate is a positive indication, as Dragendorff's reagent reacts with alkaloids to form a colored complex that precipitates out of the solution (Omotayo et al. 2022).

### 2.7 Test for Flavonoid

To determine the presence of flavonoids in the mango seed extract (MSE), a qualitative chemical test was performed. The extract was initially mixed with a few drops of diluted sodium hydroxide (NaOH). The formation of yellow‐colored precipitates indicated a positive result for flavonoids. This color change is due to the reaction between flavonoids and NaOH, which forms a colored salt. To confirm the presence of flavonoids, diluted hydrochloric acid (HCl) was subsequently added to the mixture. The disappearance (or becoming colorless) of the yellow precipitates upon the addition of HCl further confirmed the existence of flavonoids in the MSE. This is because HCl neutralizes the alkaline conditions, disrupting the flavonoid‐NaOH complex and causing the color to fade.

RETRACTED

### 2.8 Test for Tannin

To assess the presence of tannins in the mango seed extract (MSE), a ferric chloride test was conducted. The extract was mixed with a few drops of ferric chloride reagent (typically a 5% solution of FeCl_3_ in water). The observation of a blue or greenish‐black precipitate or coloration indicated the presence of tannins. This reaction occurs because tannins react with ferric ions to form colored complexes, with the specific color varying depending on the type of tannins present. The formation of a blue precipitate is generally associated with gallotannins, while a greenish‐black color indicates the presence of condensed tannins.

### 2.9 Test for Phlobatannin

To determine the presence of phlobatannins in the mango seed extract (MSE), a hydrochloric acid (HCl) precipitation test was performed. The extract was boiled with a 2 N HCl solution. The development of a red precipitate indicated the presence of phlobatannins. Phlobatannins are known to decompose upon heating in the presence of HCl, yielding a red‐colored precipitate, which serves as a positive indicator for their presence. This test is based on the property of phlobatannins to yield phlobatannin reds when depolymerized in the presence of a strong acid (Chukwudebe et al. 2019).

### 2.10 Test for Triterpene

To determine the presence of triterpenes in the mango seed extract (MSE), the Liebermann‐Burchard test, with slight modifications, was employed. A mixture of the extract and a few drops of concentrated sulfuric acid (H_2_SO_4_) was carefully prepared. The formation of a red‐brown ring at the interface between the extract and the acid layer indicated the presence of triterpenes. This reaction is based on the ability of triterpenes to undergo dehydration and cyclization in the presence of a strong acid, resulting in the formation of colored products that concentrate at the interface. It is crucial to add sulfuric acid slowly and carefully to avoid excessive heat generation, which could interfere with the reaction.

### 2.11 Test for Steroid

To determine the presence of steroids in the mango seed extract (MSE), the Liebermann‐Burchard reaction was performed. The extract was initially mixed with 2 mL of acetic anhydride in a clean, dry test tube. Subsequently, 2–3 drops of concentrated sulfuric acid (H_2_SO_4_) were carefully added down the side of the test tube, allowing it to form a distinct layer beneath the extract‐acetic anhydride mixture. The development of a blue–green ring at the interface between the two layers indicated the presence of steroids. This reaction is based on the ability of steroids to undergo dehydration and oxidation in the presence of acetic anhydride and sulfuric acid, leading to the formation of colored products. The Liebermann‐Burchard reaction is a classical test for steroids and is sensitive to the presence of a steroidal nucleus. Care was taken to ensure anhydrous conditions for optimal results.

RETRACTED

### 2.12 Test for Saponin

To assess the presence of saponins in the mango seed extract (MSE), a froth formation test was conducted. A known quantity of the extract was mixed with 5 mL of distilled water in a test tube. The mixture was then vigorously shaken for approximately 30 s to create a homogenous dispersion. Subsequently, the test tube was heated gently for a few minutes (e.g., in a water bath at 60°C for 5 min) to enhance saponin solubility and promote froth formation. After heating, the mixture was allowed to stand undisturbed for 15 min. The formation of a stable froth layer, typically 1–2 cm in height, that persisted for at least 15 min indicated the presence of saponins. Saponins are known for their ability to form stable soapy froths in aqueous solutions due to their amphipathic nature, which allows them to reduce surface tension. The height and stability of the froth are indicative of the saponin concentration in the extract.

### 2.13 FTIR Spectroscopy

The powder of MSE was evaluated in a triplicate manner to obtain FTIR spectra by KBr disc. For this, crude powder of the drug (1 mg) and KBr (100 mg) were mixed and then the resultant mixture was shifted into the die that was compressed by a hydraulic press to get the disc to get FTIR spectra in the range of 4000–400 cm^−1^. This disc was utilized to attain the results (Donga and Chanda 2021).

### 2.14 DPPH Free Radical Scavenging Assay

The DPPH radical scavenging activity of the extract was determined by a method (Huang et al. 2018). DPPH radical absorbed maximum at 517 nm against the blank solution, which disappears due to reduction by antioxidant micro compounds present in the extract. To find out the scavenging activity of the extract (10–150 μg/mL) was added to 3 mL of 1 mM DPPH solution in methanol. The whole mixture was shaken and kept in the dark at room temperature for 30 min. As a positive reference, ascorbic acid was used. The complete experiment was carried out in triplicate. The percentage inhibition of DPPH free radical scavenging capacity was calculated by the following Equation (1).

(1) $$\text{Inhibition}\;\left(\%\right)=\frac{\left(A‐\text{Blank}-A‐\text{Extract}\right)}{\;A‐\text{blank}}*100,$$

where A‐Blank: absorbance of DPPH solution with methanol, and A‐Extract: absorbance of DPPH solution with the extract.

RETRACTED

### 2.15 Nitric Oxide Scavenging Method

Sodium nitroprusside is a prerequisite to produce nitric oxide. At physiological pH, nitric oxide releases nitric acid that converts into nitrous acid, which finally produces the nitrite ion. This nitrite ion diazotizes with sulphanilic acid, which upon coupling with naphthyl‐ethylenediamine produces a pink color (Griess reagent) that can be assessed at 546 nm. The extract at a concentration of 100 μg/mL was incubated with sodium nitroprusside and phosphate buffer for 30 min at 25°C. The solution (0.5 mL) was incorporated with 1 mL of Griess reagent, incubated, and the absorbance was noted (Bernal‐Mercado et al. 2018).

The following Equation (2) was used for the calculation of nitric oxide radical scavenging potential.

(2) $$\text{Inhibition}\;\left(\%\right)=\frac{A_{c}-A_{e}}{A_{c}}*100,$$

where *A*_*c*_ was the absorbance of the control (without extract), and *A*_*e*_ was the absorbance with MSE.

### 2.16 Animal Ethical Committee

The study was started after receiving approval for the study design from the Institutional Review Board of Government College University, Faisalabad, bearing reference no. GCUF/IRB/2082.

### 2.17 Cytotoxicity Assay

According to the guidance given by the ATCC, the human hepatocellular carcinoma cell line (HepG2) was preserved. The HepG2 cell line was cultured in 10% fetal bovine serum and 0.1% streptomycin. Under the atmosphere containing CO_2_ (5%) in a humidified incubator, these cells were incubated and subcultured at the preconfluent densities by try‐EDTA (0.25%). The MTT analysis was performed to evaluate the cytotoxic potential of MSE. The 96‐well plate was utilized for the growth of cells at a density of 5 × 10^4^ cells per plate. After a 24‐h incubation period, the cells were treated with different sample concentrations and given another 48‐h incubation period. After the addition of MTT solution (25 μL of 5 mg/mL, Roche) to each well, the plates were reincubated for 4 h. The DMSO (100 μL) was added to solubilize the formed formazan crystals. The medium was removed, and the total amount of formazan crystal was measured using the spectrophotometer at an absorbance of 940 nm. The IC_50_ value for all the constituents was calculated.

### 2.18 GC–MS Analysis of MSE

Characterization of the sample was carried out through GC–MS (Shimadzu QP2010, MS Detector SPD 20A). The column Agilent (HP‐5MS, 30 m × 250 μm 0.25 μm) was packed with 5% phenyl methyl siloxane as a stationary phase. As a mobile phase, helium gas was used. Initially, the temperature was at 50°C for at least 3 min, and then it was increased to 10°C–18°C for 15 min. In the second phase, the temperature was increased to 300°C, and the pressure and temperature of the oven were recorded as 9.05 psi and 360°C, respectively. The run‐up time was 68 min, and the mass spectra obtained were matched with data available in Replib and Mainlib. The electron impact is used as the source of ionization at 250°C (Farooq et al. 2019).

RETRACTED

### 2.19 Molecular Dynamics Simulations (MDS)

Computer simulation can be expressed as a virtual laboratory. The MDS technique has been extensively used to explore the structural evolution and corresponding properties of plant bio‐constituents at the microscopic scale. MDS was performed by Schrödinger LLC Desmond software for 100 ns (Bowers et al. 2006). Protein and ligand docking were executed as the first critical step before MD modeling to define the static viewpoint of the molecule's binding location at the target's active site (Ferreira et al. 2015). Usually, MD models forecast the ligand‐binding state within a physiological setting and reproduce the movements of atoms across time (Hildebrand et al. 2019; Rasheed et al. 2021). The ligand–receptor complex (ligand: thiazole; against A: estrogen_receptor_beta_9256 and B: Progesteron_9256) and the system constructed by the System Builder tool were optimized, minimized, and replaced with missing residues using Maestro's Protein Preparation Wizard. The OPLS_2005 force field, 310 K temperature, and 1 atm pressure were used in the TIP3P (Intermolecular Interaction Potential 3 Points Transferable) fluid model (Shivakumar et al. 2010). To mimic physiological conditions during the neutralization of the models, 0.15 M NaCl with neutralizing ions was utilized. Models were released before modeling, and pathways were stored for inspection every 100 ps.

### 2.20 Toxicological Evaluation

The study was performed after getting approval for the study design from the Institutional Review Board of the Government College University, Faisalabad, bearing reference no. GCUF/IRB/2082.

### 2.21 Subacute Oral Toxicity Assay

A subacute toxicity study was executed on nulliparous, non‐pregnant Wistar rats of both sexes (7–11 weeks) weighing 165–200 g, selected randomly. They were retained in standard laboratory conditions at a temperature (23°C ± 2°C), a 12‐h light/dark cycle, humidity 35%–65%, fed a normal pellet diet and water ad libitum about 1 week before the commencement of the experiment. The selection of dose levels was based on results attained from the acute toxicity study (OECD 423 guidelines) that had already been performed (Villas‐Boas et al. 2021). The dose was calculated according to body weight. Subacute toxicity analysis was performed following OECD guideline 407 (Dawud et al. 2023). The animals were assorted into four groups. Group I: served as a negative control receiving distilled water (1 mg/kg). Group II–IV: Treated with different (250, 500 and 1000 mg/mL) doses of MSE orally for 28 days.

RETRACTED

Clinical examination, water and food intake, gain in body weight, and any signs and symptoms of toxicity were observed. Close observation for clinical signs and symptoms was made for the first 30 min, then for the next 4 h, and once a day regularly up to 28 days. Food was administered after a few hours of dosing. Both the negative control group (*n* = 6) and the MSE‐treated groups received a similar amount of distilled water (Figure 1). In the last part of the observational period, all surviving rats were weighed, and blood samples were taken through cardiac puncture under ether anesthesia for analysis of biochemical and hematological biomarkers. The vital organs were removed and weighed after the assassination of the rats through cervical dislocation and kept for histopathological examination in 10% formalin.

**FIGURE 1:** Timeline diagram of MSE for evaluation of oral subacute toxicity.

### 2.22 Biochemical Analysis

Lipid profiles, including total cholesterol, HDL, triglycerides, and LDL, were determined according to the methods described by several authors (Richmond 1973; Allain et al. 1974; Lopes‐Virella et al. 1977; Fossati and Prencipe 1982; Wieland and Seidel 1983), respectively. Colorimetric assays were used to measure alanine aminotransferase (ALT), aspartate aminotransferase (AST), and alkaline phosphatase (ALP) spectrophotometrically (Fossati and Prencipe 1982; Wieland and Seidel 1983). Total bilirubin was determined using spectrophotometry. Total protein (TP) and albumin levels were evaluated by using the method mentioned in Lee and Gartner (1976). Globulin was determined using the method described by Chary and Sharma (2004). All the quantitative measurements were conducted using spectrophotometric kits (Biodiagnostic Company, UK). Biochemical parameters were measured in blood samples collected from each animal. Serum and plasma were separated through centrifugation using a Sigma Laboratories, GMBH, West Germany, model 2‐153360 Osterode/Hz centrifuge operating at 4000 g/min for 15 min (Poomanee et al. 2021).

### 2.23 Blood Parameters

The hematological parameters, including hemoglobin (HB), red blood cell count (RBC), white blood cell count (WBC), neutrophils, lymphocytes, monocytes, and eosinophils, were assessed using an automated hematology analyzer (XT‐2000iv, SYSMEX Co. Ltd., Kobe, Japan) (George et al. 2019).

RETRACTED

### 2.24 Histopathological Examination

The isolated vital organs (heart, liver, and kidney) were initially preserved in 10% formalin after the processing step and then set in paraffin wax. A tissue section (5 mm) was taken and stained with hematoxylin and eosin. The required tissue structure was placed below a light microscope for examination (RamPravinKumar and Dhananjayan 2021).

### 2.25 Statistical Analysis

All data were expressed as the mean ± standard deviation (SD) of triplicate measurements. Statistical significance was determined using one‐way ANOVA followed by Tukey's post hoc test. A *p*‐value of less than 0.05 was considered statistically significant. Statistical analyses were performed using SPSS (version 29). Dose–response curves and IC_50_ values were calculated using the non‐linear regression analysis within Microsoft Excel. Figures were generated using GraphPad Prism and Microsoft Excel.

## 3 Results

### 3.1 Nutritional Composition and Mineral Analysis of Mango Seed Extract (MSE)

The obtained results of the nutritional analysis of MSE revealed that it contains crude protein (8.5% ± 0.01%), oil (13.5% ± 0.06%) and fiber (2.8% ± 0.02%), carbohydrate (35% ± 0.01%), ash (1.8% ± 0.05%), and 405 kJ/100 g of energy content. The analysis of the MSE for mineral content indicates the presence of macrominerals in the following order: K > Mg > P > Ca > Na. The mineral analysis of MSE indicated magnesium (24.5 ± 2.54 mg/100 g dry), phosphorus (21.0 ± 1.36 mg/100 g dry), calcium (9.80 ± 3.65 mg/100 g dry), and sodium (2.44 ± 1.65 mg/100 g dry), respectively.

### 3.2 Amino Acid and Vitamin Content

The amino acid and vitamin profiles of mango seed extract (MSE), as presented in Table 1, underscore its nutritional value. Among essential amino acids, MSE contains notable amounts of valine (3.59 ± 2.65 mg/100 g), threonine (1.99 ± 2.45 mg/100 g), methionine (6.98 ± 3.69 mg/100 g), lysine (3.21 ± 1.23 mg/100 g), histidine (2.56 ± 1.54 mg/100 g), and cysteine (2.30 ± 4.23 mg/100 g). The nonessential amino acids identified include tyrosine (3.39 ± 3.65 mg/100 g), serine (2.58 ± 1.22 mg/100 g), proline (2.89 ± 1.56 mg/100 g), leucine (8.30 ± 5.23 mg/100 g), isoleucine (3.14 ± 1.54 mg/100 g), glycine (3.14 ± 2.33 mg/100 g), and glutamate (12.8 ± 2.16 mg/100 g).

**TABLE 1:** Amino acid composition and vitamin content of MSE (mg/100 g of protein).

Amino acids	Value
Essential amino acids	
Valine	3.59 ± 2.65
Threonine	1.99 ± 2.45
Methionine	6.98 ± 3.69
Lysine	3.21 ± 1.23
Histidine	2.56 ± 1.54
Cysteine	2.30 ± 4.23
Aspartate	3.58 ± 1.25
Arginine	5.30 ± 2.25
Alanine	5.90 ± 2.11
Nonessential amino acids	
Tyrosine	3.39 ± 3.65
Serine	2.58 ± 1.22
Proline	2.89 ± 1.56
Leucine	8.30 ± 5.23
Isoleucine	3.14 ± 1.54
Glycine	3.14 ± 2.33
Glutamate	12.8 ± 2.16
Vitamins (mg/100 g)	
A	14.9 ± 1.32
C	4.65 ± 0.58
E	3.65 ± 1.40
K	2.39 ± 0.61

*Note:* Each experiment was performed in triplicate (mean ± SD).

RETRACTED

Regarding vitamin content, MSE is a source of vitamin A (14.9 ± 1.32 mg/100 g), vitamin C (4.65 ± 0.58 mg/100 g), vitamin E (3.65 ± 1.40 mg/100 g), and vitamin K (2.39 ± 0.61 mg/100 g). All measurements were performed in triplicate and are reported as mean ± standard deviation, highlighting MSE's potential as a valuable ingredient rich in essential amino acids and vitamins for health and nutrition applications.

### 3.3 Phytochemical Analysis

Table 2 presents the qualitative phytochemical evaluation of MSE, highlighting the presence and abundance of various phytochemicals. The analysis revealed the following results: alkaloids were identified using Dragendroff's test, indicating their presence (+); flavonoids were detected with an alkaline reagent, also confirming their presence (+). Tannins showed a strong positive result in the FeCl_3_ test, indicating a high concentration (+++). In contrast, phlobatannins were not detected using the HCl test (−), whereas triterpenes were moderately present as indicated by the H_2_SO_4_ test (++). Steroids were absent according to the Liebermann‐Burchard test (−), and saponins were also not detected in the frothing test (−).

**TABLE 2:** Qualitative phytochemical evaluation of MSE.

Phytochemicals identified	Name of chemical test	Inference
Alkaloids	Dragendroff's test	+
Flavonoids	Alkaline reagent	+
Tannins	FeCl_3_ test	+++
Phlobatannins	HCl test	−
Triterpene	H_2_SO_4_ test	+++
Steroids	Liebbermann‐burchard test	−
Saponins	Frothing test	−

*Note:* The results are summarized with an inference scale where absence is denoted as “−,” trace as “+,” moderate presence as “++,” and excellent presence as “+++,” illustrating the diverse phytochemical profile of MSE and its potential health benefits.

### 3.4 DPPH Free Radical and Nitric Oxide Scavenging Property

Figure 2 summarizes the antioxidant activity of MSE compared to ascorbic acid, a well‐known antioxidant. The methanolic extract of MSE demonstrated potent antioxidant activity, as evidenced by its high DPPH radical scavenging capacity, with an inhibition percentage of 95.86% ± 2.31%. This activity exceeded that of the standard antioxidant, ascorbic acid, which exhibited 92.55% ± 4.70% inhibition. Furthermore, MSE also displayed substantial nitric oxide (NO) scavenging activity, with an inhibition rate of 89.36% ± 5.25%, surpassing that of ascorbic acid, which recorded 80.45% ± 4.12% inhibition. These results, expressed as mean ± standard error of the mean (SEM; *n* = 3), underscore the strong antioxidant potential of MSE. The pronounced free radical scavenging activity suggests its promising application as a natural antioxidant in health and nutrition, potentially contributing to its observed pharmacological properties.

RETRACTED

**FIGURE 2:** Antioxidant activity of MSE.

### 3.5 FTIR Analysis

The FTIR analysis of the MSE was conducted to identify key phytochemicals in the sample. The qualitative standardization revealed several significant spectral peaks, indicating the presence of various functional groups. Notably, peaks corresponding to N–H bonds were observed at 3853.85 and 3750.39 cm^−1^, whereas O–H bonds were identified at 3649.25 and 3275.17 cm^−1^, suggesting the presence of amines and alcohols. The C–H alkane groups were detected at 2917.38 and 2849.43 cm^−1^, indicating saturated hydrocarbons. Additionally, a peak for the C=O conjugated aldehyde was noted at 1699.16 cm^−1^, and C=N imine/oxime was present at 1647.68 cm^−1^. The analysis also identified nitro compounds (N–O) at 1541.53 and 1456.52 cm^−1^, as well as cyanide (C–N) functional groups at multiple wavelengths (1338.68, 1203.12, 1150.31, and 1075.68 cm^−1^). Last, methene (=C–H) groups were detected at 996.83 and 861.60 cm^−1^. These findings, illustrated in Figure 3, provide a comprehensive fingerprint of the phytochemical profile of MSE, highlighting its potential health benefits and applications in various fields such as nutrition and pharmacology.

**FIGURE 3:** FTIR analysis of crude powder of MSE.

### 3.6 Screening of Cytotoxic Effect of MSE

The MTT viability assay was utilized to assess the cytotoxic potential of MSE against the HePG2 cell line. Cells were incubated with varying concentrations of MSE (ranging from 12.5 to 200 μg/mL) for 24–48 h, and cell growth was evaluated posttreatment. The results demonstrated a concentration‐dependent cytotoxic effect, with the highest concentration of 200 μg/mL exhibiting a maximum cytotoxicity of 48.5% (Figure 4A), indicating significant antitumor activity against cervical cancer cells. The IC_50_ value for MSE was determined to be 140 μg/mL, as illustrated in Figure 4B. These findings suggest that MSE possesses considerable potential as a natural anticancer agent, warranting further investigation into its mechanisms of action and therapeutic applications.

**FIGURE 4:** Bar graphs of MTT assay. (A) Cytotoxic potential and (B) IC_50_ of MSE.

RETRACTED

### 3.7 GC–MS Analysis of MSE

The GC–MS analysis of aqueous methanol extracts of MSE revealed a variety of bioactive constituents with significant phytochemical activities. The chromatogram highlights the presence of several compounds, including thiazole, 2‐ethylacridine, silicic acid, arsenous acid, 3,5‐ethanoquinolin‐10‐one, and hexahydropyridine. These identified compounds are associated with various biological actions such as antioxidant, anticancer, antiandrogenic, and anticoronary properties. Drug combinations used in adults can benefit children with acute promyelocytic leukemia. Arsenic has been used in combination with all trans retinoic acid (ATRA) for the treatment of acute promyelocytic leukemia (APL) (Liu et al. 2021). The data underscore the potential of MSE as a source of bioactive compounds that could be utilized in nutraceutical applications and further research into their therapeutic effects. The detailed chemical components, along with their molecular formulas, concentrations, retention times, and molecular weights, are summarized in Table 3. This comprehensive analysis demonstrates the diverse phytochemical profile of MSE and its potential health benefits. The chromatograph of the MSE extract is shown in Figure 5.

**TABLE 3:** List of different bioactive components present in MSE in GC–MS.

Sr. no	Area	Retention time	Compounds name	Molecular formula	Molecular weight
1	0.54	2.669	Thiazole	C_3_H_3_NH	85.13 g/mol
2	0.40	29.441	2‐Ethylacridine	C_15_H_13_N	207.02 g/mol
3	0.89	29.812	Silicic acid	H_4_O_4_Si	78.091 g/mol
4	0.94	33.150	Arsenous Acid	H_3_AsO_3_	125.02 g/mol
5	1.23	29.860	3,5‐Ethanoquinolin‐10‐one	C_13_H_21_NO	207.21 g/mol
6	0.94	33.510	Hexahydropyridine	C_12_H_17_NO_2_	193.24 g/mol

**FIGURE 5:** GC–MS analysis MSE extract.

In recent years, nutraceuticals have garnered considerable interest for their potential role in managing chronic diseases, including diabetes mellitus. While the present study primarily focused on the phytochemical composition, antioxidant capacity, and safety profile of MSE, the inclusion of literature emphasizing its broader nutraceutical implications is essential. Previous investigations have demonstrated the antidiabetic potential of mango‐derived compounds, which include improved glucose tolerance, enhanced lipid profiles, and reduced beta‐cell damage. For instance, some studies on cordycepin have provided mechanistic insights into how plant‐derived bioactives modulate metabolic pathways relevant to diabetes management (Ashraf et al. 2020; Baruah et al. 2023). Although this study did not include direct assessments of glucose uptake or enzyme inhibition, the promising cytotoxic and antioxidant properties, coupled with the presence of bioactives like flavonoids and thiazole derivatives, suggest a potential for MSE in mitigating oxidative stress‐related complications of diabetes. Future investigations will be directed toward elucidating the specific antidiabetic mechanisms of MSE through targeted assays such as α‐glucosidase inhibition, glucose uptake studies, and insulin signaling pathway analysis to substantiate its functional role as a nutraceutical.

RETRACTED

### 3.8 Molecular Dynamic Simulations (MDS)

The affinity of the ligand was evaluated through molecular docking simulations throughout 100 ns (ns), allowing for an assessment of the interaction between the ligand and the receptor. The stability of the ligand–receptor complex was monitored by analyzing time‐dependent fluctuations in the root mean square deviation (RMSD). This simulation study served as a critical preliminary step before conducting molecular dynamics (MD) simulations, as it provided insights into the static binding orientation of the molecule at the active site of the target. By establishing this foundational understanding, the study aimed to enhance the accuracy of subsequent MD analyses and further elucidate the dynamic behavior of the ligand–receptor interactions (Ferreira et al. 2015).

According to the RMSD analysis presented in Figure 6A,B, the ligand–receptor complex displayed initial stability, with some fluctuations beginning at 20 ns, where a slight increase in RMSD was noted. In contrast, the RMSD of the protein‐bound ligand exhibited stability from 10 ns onward, showing no significant variation or modification in the simulated protein–ligand fit analyses after this point. These results indicate that the compound remains stable throughout the simulation. The root mean square fluctuation (RMSF) values of the protein–ligand complex were calculated and are illustrated in Figure 6C,D. The higher peaks observed in the loop regions of the MD trajectories suggest the stability of these residues, whereas low RMSF values indicate strong binding stability of the chosen ligand to the target protein. During the simulation, secondary structure elements, including beta‐strands and alpha‐helices, were monitored. Figure 6E shows that alpha‐helices constituted 26.05% and beta‐strands 12.24% of the secondary structural elements, totaling 38.29%. In Figure 6F, these values were recorded as 31.20% for alpha‐helices and 2.62% for beta‐strands, resulting in a total of 33.82%. The ratio of beta sheets to alpha‐helices also influenced the protein's RMSD; residues within these rigid structures exhibited lower RMSD compared to those located in more flexible coils and loops. Significant ligand–protein interactions were primarily mediated by hydrogen bonds, as depicted in Figure 6G,H. The molecular contacts and interactions—encompassing hydrogen bonds, hydrophobic interactions, ionic bonds, and water bridges—demonstrated the binding affinity between the target protein and the ligand. Specifically, Figure 6I highlights hydrogen bonding involving GLU_305 residues, while hydrophobic interactions were observed with PRO_277, TRP_312, and TRP_345 residues. Additionally, Figure 6J illustrates hydrophobic bonding with LEU_715 and PHE_905 residues. Throughout the simulation analyses, critical observations of ligand–protein interactions further confirmed the stability and efficacy of the binding process.

RETRACTED

**FIGURE 6:** (A) Estrogen_receptor_beta_9256 (ER‐b) shows the RMSD between C‐alpha atoms of protein and ligand over time, (B) Progesteron_9256 (PR), differences in ligand protein RMSD shifts over time, (C, D) represent ER‐b and PR root mean square fluctuation of the target protein residues complex, (E, F) ER‐b and PR simulation shows secondary structure elements (alpha‐helix and beta‐strands) of protein, (G, H) represent the ER‐b and PR protein‐ligand contacts histogram throughout the trajectories. (I) Ligand atom interactions with the protein residues (ER‐b), (J) the schematic of detailed ligand atom interactions with the protein residues (PR).

### 3.9 Subacute Toxicity Study

#### 3.9.1 Behavioral Pattern

The administration of MSE resulted in an increased urination rate and decreased fecal consistency compared to the negative control group. Other parameters, including salivation, somatomotor activity, sleep, respiration, mortality, mucous membrane condition, skin, fur, eyes, corneal reflex, convulsions, and coma, remained unchanged between the treated and negative control groups throughout the experimental period, as detailed in Table 4. These findings suggest that while MSE may influence urinary output and fecal characteristics, it does not significantly affect other physiological parameters. This aligns with existing literature that highlights the relationship between bowel habits and urinary tract function, indicating that changes in stool consistency can impact urinary symptoms. Further investigation into the mechanisms underlying these effects is warranted to fully understand the implications of MSE for gastrointestinal and urinary health.

**TABLE 4:** Effect of MSE on treated and vehicle groups for behavioral pattern assessment in rats.

Parameters	Negative control	MSE (250 mg/mL)	MSE (500 mg/kg)	MSE (1000 mg/kg)
Coma	A	A	A	A
Convulsions	A	A	A	A
Torch pupil response	C	C	C	C
Corneal reflux	C	C	C	C
Eyes	C	C	C	C
Skin	C	C	C	C
Touch response fur	C	C	C	C
Itching	C	C	C	C
Feces consistency	C	D	D	D
Mucous membrane	C	C	C	C
Mortality	C	C	C	C
Respiration	C	C	C	C
Somatomotor activity and behavior pattern	C	C	C	C
Sleep	C	C	C	C
Salivation	C	C	C	C
Urination	I	I	I	I

*Note:* Values are presented as means ± SD (*n* = 6).

RETRACTED

Abbreviations: A, absent; C, common (normal); D, decrease; I, increase.

#### 3.9.2 Body Weight and Index of the Organ to Body Weight

The data presented in Table 5 illustrate the effects of MSE on body weight and food and water consumption in treated rats compared to a negative control group. The initial weights of the rats showed nonsignificant differences among the groups, with the negative control at 199.3 ± 1.20 g, while MSE‐treated groups recorded initial weights of 194.1 ± 2.08 g (250 mg/kg), 198.3 ± 1.76 g (500 mg/kg), and 202.6 ± 1.20 g (1000 mg/kg). At the end of the study, final weights were also similar across groups, with the negative control at 203 ± 1.52 g and MSE‐treated groups showing final weights of 199.3 ± 2.33 g (250 mg/kg), 205.1 ± 1.15 g (500 mg/kg), and 207.6 ± 1.45 g (1000 mg/kg), again indicating nonsignificant differences. Food intake was slightly lower in all MSE‐treated groups compared to the negative control group, with values of 112 ± 2.08 g/day (250 mg/kg), 114.6 ± 2.60 g/day (500 mg/kg), and 113.6 ± 1.20 g/day (1000 mg/kg) versus the control's intake of 116.1 ± 1.15 g/day, although these differences were also nonsignificant. Water intake showed minor variations as well, with MSE‐treated groups consuming between 195.1 ± 1.73 mL/day (500 mg/kg) and 200 ± 1.52 mL/day (1000 mg/kg) compared to the negative control's consumption of 194 ± 1.15 mL/day, all classified as nonsignificant compared with the negative control group. Overall, these findings suggest that MSE treatment does not significantly affect body weight or food and water consumption in rats at the administered doses.

**TABLE 5:** Effect of MSE in treated and vehicle groups on body weight and consumption of food and water in rats.

Parameters	Negative control	MSE (250 mg/kg)	MSE (500 mg/kg)	MSE (1000 mg/kg)	*p*
Initial weight (g)	199.3 ± 1.20^a^	194.1 ± 2.08^a^	198.3 ± 1.76^a^	202.6 ± 1.20^a^	0.12^NS^
Final weight (g)	203 ± 1.52^a^	199.3 ± 2.33^a^	205.1 ± 1.15^a^	207.6 ± 1.45^a^	0.34^NS^
Intake of food (g/day)	116.1 ± 1.15^a^	112 ± 2.08^a^	114.6 ± 2.60^a^	113.6 ± 1.20^a^	0.11^NS^
Intake of water (mL/day)	194 ± 1.15^a^	197.1 ± 1.15^a^	195.1 ± 1.73^a^	200 ± 1.52^a^	0.29^NS^

*Note:* Values are presented as means ± SD (*n* = 6).

Abbreviations: MSE, *Mangifera indica* seeds extract; NS, nonsignificant compared with negative control. ^a^Means with different superscripts indicating the level of significant difference (*p* ≤ 0.05).

RETRACTED

The organ‐to‐body weight ratios of the liver, kidney, and heart in rats treated with various doses of mango seed extract (MSE) are presented in Table 6. Across all treatment groups (250, 500, and 1000 mg/kg), there were no statistically significant differences in organ‐to‐body weight ratios compared to the negative control group for any organ examined. Specifically, liver ratios ranged from 3.53 ± 1.10 to 4.30 ± 1.45 in MSE‐treated groups versus 3.70 ± 0.11 in controls. Kidney ratios varied between 2.60 ± 0.38 and 3.60 ± 0.38 in treated groups compared to 3.01 ± 0.36 in controls. Heart ratios ranged from 1.56 ± 0.21 to 4.66 ± 0.35 in treated groups, whereas the control was 2.35 ± 0.35.

**TABLE 6:** Influence of MSE on the organ‐to‐body weight ratio in extract‐treated and vehicle‐treated groups of rats.

Organs	Negative control	MSE (250 mg/kg)	MSE (500 mg/kg)	MSE (1000 mg/kg)	*p*
Liver	3.70 ± 0.11^a^	4.30 ± 1.45^a^	3.53 ± 1.10^a^	3.96 ± 1.60^a^	0.10^NS^
Kidney	3.01 ± 0.36^a^	2.65 ± 0.33^a^	2.60 ± 0.38^a^	3.60 ± 0.38^a^	0.16^NS^
Heart	2.35 ± 0.35^a^	4.66 ± 0.35^a^	1.56 ± 0.21^a^	4.22 ± 0.33^a^	0.11^NS^

*Note:* Values are presented as means ± SD (*n* = 6).

Abbreviations: MSE, *Mangifera indica* seeds extract; NS, nonsignificant compared with negative control. ^a^Means with different superscripts indicating the level of significant difference (*p* ≤ 0.05).

These findings indicate that oral administration of MSE at doses up to 1000 mg/kg does not induce significant changes in the relative weights of the liver, kidney, or heart, suggesting the absence of overt organ toxicity or hypertrophy. This supports the safety profile of MSE and aligns with the histopathological observations, further confirming that MSE does not adversely affect major organ systems at the tested doses.

#### 3.9.3 Biochemical Analysis

Table 7 presents the effects of MSE on various parameters of liver function tests in treated and vehicle groups of rats. The results indicate that the levels of alanine aminotransferase (ALT) were 204.6 ± 2.02 U/L in the negative control group, with MSE‐treated groups showing values of 205.6 ± 2.02 U/L (250 mg/kg), 208.6 ± 1.20 U/L (500 mg/kg), and 204.6 ± 2.02 U/L (1000 mg/kg). All results indicate a nonsignificant effect of all treatments compared with negative control. Similarly, aspartate aminotransferase (AST) levels were recorded at 334 ± 1.73 U/L for the negative control, with MSE treatments resulting in values of 334.6 ± 1.45 U/L (250 mg/kg), 337 ± 1.15 U/L (500 mg/kg), and 335.0 ± 1.15 U/L (1000 mg/kg), also showing nonsignificant differences. The alkaline phosphatase (ALP) levels were similar, with the negative control at 161.3 ± 1.45 U/L and MSE‐treated groups showing values of 162.6 ± 1.45 U/L (250 mg/kg), 160.6 ± 1.20 U/L (500 mg/kg), and 161.6 ± 1.85 U/L (1000 mg/kg), all classified as nonsignificant.

RETRACTED

**TABLE 7:** Effect of MSE‐treated and vehicle groups on parameters of liver function tests in rats.

Parameters	Negative control	MSE (250 mg/kg)	MSE (500 mg/kg)	MSE (1000 mg/kg)	*p*
ALT (U/L)	204.6 ± 2.02^a^	205.6 ± 2.02^a^	208.6 ± 1.20^a^	204.6 ± 2.02^a^	0.61^NS^
AST (U/L)	334 ± 1.73^a^	334.6 ± 1.45^a^	337 ± 1.15^a^	335.0 ± 1.15^a^	0.54^NS^
ALP (U/L)	161.3 ± 1.45^a^	162.6 ± 1.45^a^	160.6 ± 1.20^a^	161.6 ± 1.85^a^	0.48^NS^
Bilirubin (mg/dL)	1.14 ± 0.76^a^	1.11 ± 0.80^a^	2.14 ± 0.96^b^	1.15 ± 0.60^a^	0.26^NS^
Total protein (G/dL)	6.83 ± 1.17^a^	6.76 ± 2.17^a^	6.90 ± 1.23^a^	6.76 ± 2.14^a^	0.32^NS^
Albumin (G/dL)	4.26 ± 2.14^a^	4.36 ± 2.18^a^	3.90 ± 2.11^a^	4.13 ± 3.20^a^	0.19^NS^
Globulin (G/dL)	2.16 ± 1.14^a^	2.53 ± 1.12^a^	2.20 ± 3.17^a^	2.70 ± 1.17^a^	0.22^NS^

*Note:* Values are presented as means ± SD (*n* = 6).

Abbreviations: MSE, *Mangifera indica* seeds extract; NS, nonsignificant compared with negative control. ^a^Means with different superscripts indicating the level of significant difference (*p* ≤ 0.05).

Bilirubin levels were slightly elevated in MSE‐treated groups, with the negative control at 1.14 ± 0.76 mg/dL compared to MSE treatments of 1.11 ± 0.80 mg/dL (250 mg/kg), 2.14 ± 0.96 mg/dL (500 mg/kg), and a decrease to 1.15 ± 0.60 mg/dL (1000 mg/kg); however, these changes were not statistically significant either. Total protein levels remained consistent across groups, with the negative control at 6.83 ± 1.17 g/dL and MSE‐treated groups at 6.76 ± 2.17 g/dL (250 mg/kg), 6.90 ± 1.23 g/dL (500 mg/kg), and again at 6.76 ± 2.14 g/dL (1000 mg/kg). Albumin levels were similar across groups, showing values of 4.26 ± 2.14 g/dL for the negative control and ranging from 3.90 ± 2.11 to 4.36 ± 2.18 g/dL in MSE‐treated groups, whereas globulin levels showed a slight increase in treated groups but remained nonsignificant overall. These findings suggest that MSE treatment does not significantly affect liver function parameters in rats at the tested doses, indicating a favorable safety profile for the extract regarding hepatic health, as presented in Table 7.

#### 3.9.4 Lipid Profile

Table 8 outlines the effect of MSE on the lipid profile of the treated and vehicle groups of rats. The cholesterol levels in the negative control group were recorded at 162.3 ± 1.45 mg/dL, whereas MSE‐treated groups exhibited lower cholesterol levels: 160.3 ± 2.02 mg/dL (250 mg/kg), 150.1 ± 2.80 mg/dL (500 mg/kg), and 144.3 ± 2.40 mg/dL (1000 mg/kg), with all differences being significant compared to the negative control. High‐density lipoprotein (HDL) levels showed an increase in MSE‐treated groups, starting from 32 ± 1.15 mg/dL in the negative control to 35.3 ± 1.20 mg/dL (250 mg/kg), 44.6 ± 1.45 mg/dL (500 mg/kg), and 48.2 ± 1.15 mg/dL (1000 mg/kg), indicating a potential positive effect on HDL levels, though these changes were highly significant, as described in Table 8.

RETRACTED

**TABLE 8:** Effect of MSE in treated and vehicle groups on lipid profile in rats.

Parameters	Negative control	MSE (250 mg/kg)	MSE (500 mg/kg)	MSE (1000 mg/kg)	*p*
Cholesterol (mg/dL)	162.3 ± 1.45^a^	160.3 ± 2.02^a^	150.1 ± 2.80^b^	144.3 ± 2.40^c^	0.03*
HDL (mg/dL)	32 ± 1.15^d^	35.3 ± 1.20^c^	44.6 ± 1.45^b^	48.2 ± 1.15^a^	0.01**
LDL (mg/dL)	112.2 ± 1.17^a^	104.6 ± 1.45^b^	98.1 ± 1.18^c^	95.3 ± 3.88^d^	0.04*
Triglyceride (mg/dL)	123.1 ± 1.13^a^	120.6 ± 1.20^b^	111.6 ± 1.70^c^	106.3 ± 1.76^d^	0.01**
VLDL (mg/dL)	24.6 ± 1.45^a^	20.3 ± 2.88^b^	17.3 ± 1.20^c^	11.6 ± 1.76^d^	0.02*

*Note:* Values are presented as means ± SD (*n* = 6). ^a–d^Means with different superscripts showing statistically significant difference (*p ≤* 0.05), **p ≤ 0.01, and *p ≤ 0.05.

Abbreviation: MSE, *Mangifera indica* seeds extract.

Low‐density lipoprotein (LDL) levels were measured at 112.2 ± 1.17 mg/dL for the negative control, with MSE treatments resulting in values of 104.6 ± 1.45 mg/dL (250 mg/kg), 98.1 ± 1.18 mg/dL (500 mg/kg), and 95.3 ± 3.88 mg/dL (1000 mg/kg), showing a significant difference across groups. Triglyceride levels were slightly reduced in the MSE‐treated groups, with values of 120.6 ± 1.20 mg/dL (250 mg/kg), 111.6 ± 1.70 mg/dL (500 mg/kg), and 106.3 ± 1.76 mg/dL (1000 mg/kg) compared to the negative control at 123.1 ± 1.13 mg/dL, but these variations were also classified as highly significant. Finally, very low‐density lipoprotein (VLDL) levels decreased from the negative control's value of 24.6 ± 1.45 mg/dL to lower levels in the MSE‐treated groups: 20.3 ± 2.88 mg/dL (250 mg/kg), 17.3 ± 1.20 mg/dL (500 mg/kg), and significantly reduced to 11.6 ± 1.76 mg/dL (1000 mg/kg). While these findings suggest potential benefits of MSE on lipid profiles, all results were statistically significant when compared with the negative control group, as presented in Table 8.

#### 3.9.5 Renal Profile

Table 9 summarizes the influence of MSE on renal function parameters in treated and vehicle control groups of rats. The creatinine levels in the negative control group were recorded at 2.77 ± 0.60 mg/dL, whereas MSE‐treated groups showed values of 2.11 ± 0.70 mg/dL (250 mg/kg), 3.17 ± 0.61 mg/dL (500 mg/kg), and 2.14 ± 0.46 mg/dL (1000 mg/kg). All differences were classified as nonsignificant compared to the negative control. Urea levels were similarly assessed, with the negative control group at 22.30 ± 1.45 mg/dL and MSE‐treated groups showing values of 22.00 ± 1.73 mg/dL (250 mg/kg), 18.60 ± 2.80 mg/dL (500 mg/kg), and 21.00 ± 1.15 mg/dL (1000 mg/kg), with these variations also deemed nonsignificant. These findings suggest that MSE treatment does not significantly affect renal function parameters such as creatinine and urea levels in rats at the tested doses, indicating a favorable safety profile for the extract concerning kidney health.

RETRACTED

**TABLE 9:** Influence of MSE in treated and vehicle groups on the parameter of renal function in rats.

Parameters	Negative control	MSE (250 mg/kg)	MSE (500 mg/kg)	MSE (1000 mg/kg)	*p*
Creatinine (mg/dL)	2.77 ± 0.60^a^	2.11 ± 0.70^a^	3.17 ± 0.61^a^	2.14 ± 0.46^a^	0.17^NS^
Urea (mg/dL)	22.30 ± 1.45^a^	22.00 ± 1.73^a^	18.60 ± 2.80^b^	21.00 ± 1.15^a^	0.35^NS^

*Note:* Values are presented as means ± SD (*n* = 6).

Abbreviations: MSE, *Mangifera indica* seeds extract; NS, non‐significant compared with negative control. ^a‐b^Means with different superscripts indicating the level of significant difference (*p* ≤ 0.05).

#### 3.9.6 Blood Parameters

Table 10 presents the influence of MSE on the blood analysis of treated and vehicle control groups of rats. The hemoglobin (Hb) levels in the negative control group were recorded at 5.33 ± 2.88 g/dL, whereas MSE‐treated groups showed significantly higher levels: 7.6 ± 1.20 g/dL (250 mg/kg), 9.3 ± 2.02 g/dL (500 mg/kg), and 11 ± 2.08 g/dL (1000 mg/kg), producing a significant rise compared to the negative control. The platelet count was slightly elevated in MSE‐treated groups, with values of 254.6 ± 2.60 × 10^3^/μL (250 mg/kg), 263.6 ± 2.02 × 10^3^/μL (500 mg/kg), and 274.3 ± 2.33 × 10^3^/μL (1000 mg/kg), compared to the negative control at 247.6 ± 1.45 × 10^3^/μL, but these differences were also statistically significant, as described in Table 10.

**TABLE 10:** Influence of MSE on hematological profile in treated and vehicle groups of rats.

Parameters	Negative control	MSE (250 mg/kg)	MSE (500 mg/kg)	MSE (1000 mg/kg)	*p*
Hb (g/dL)	5.33 ± 2.88^d^	7.6 ± 1.20^c^	9.3 ± 2.02^b^	11 ± 2.08^a^	0.03*
Platelet count (×10^3^/μL)	247.60 ± 1.45^d^	254.60 ± 2.60^c^	263.60 ± 2.02^b^	274.30 ± 2.33^a^	0.02*
W.B.C count (×10^3^/μL)	2.40 ± 1.11^d^	3.80 ± 1.11^c^	6 ± 2.28^b^	7.13 ± 2.17^a^	0.04*
Neutrophils (%)	8.10 ± 1.15^d^	10 ± 1.15^c^	14.00 ± 1.15^b^	20.00 ± 1.15^a^	0.03*
Lymphocytes (%)	86 ± 1.15^c^	86.6 ± 1.45^c^	91.30 ± 1.85^b^	98.60 ± 2.02^a^	0.04*
Monocytes (%)	5 ± 1.15^c^	5.33 ± 2.88^c^	7 ± 1.15^b^	9 ± 1.15^a^	0.02*
Eosinophils (%)	1.26 ± 0.37^a^	0.80 ± 0.11^a^	1.26 ± 0.37^a^	0.70 ± 0.11^a^	0.16^NS^

*Note:* Values are presented as means ± SD (*n* = 6). ^a–d^Means with different superscripts showing statistically significant difference (*p ≤* 0.05), *p ≤ 0.05.

RETRACTED

Abbreviations: MSE, *Mangifera indica* seeds extract; NS, nonsignificant compared with negative control.

The white blood cell (WBC) count in the negative control group was measured at 2.40 ± 1.11 × 10^3^/μL, with MSE treatments resulting in counts of 3.80 ± 1.11 × 10^3^/μL (250 mg/kg), 6 ± 2.28 × 10^3^/μL (500 mg/kg), and 7.13 ± 2.17 × 10^3^/μL (1000 mg/kg), indicating a significant increase in WBC count compared to the control group. Neutrophil percentages rose from 8.10% ± 1.15% in the negative control to values of 10% ± 1.15% (250 mg/kg), 14% ± 1.15% (500 mg/kg), and 20.00% ± 1.15% (1000 mg/kg), while lymphocyte percentages remained relatively stable, with the negative control at 86% ± 1.15% and MSE‐treated groups showing values of 86.60% ± 1.45% (250 mg/kg), 91.30% ± 1.85% (500 mg/kg), and increasing to 98.60% ± 2.02% (1000 mg/kg).

Monocyte percentages were consistent across groups, starting at 5% ± 1.15% for the negative control and showing slight increases in MSE‐treated groups: 5.33% ± 2.88% (250 mg/kg), 7% ± 1.15% (500 mg/kg), and reaching up to 9% ± 1.15% (1000 mg/kg). Eosinophil percentages varied slightly, with the negative control at 1.26% ± 0.37%, while MSE‐treated groups showed values of 0.80% ± 0.11% (250 mg/kg), maintaining approximately similar levels for higher doses. Overall, these findings indicate that MSE treatment may influence certain hematological parameters, particularly hemoglobin and WBC counts, although all results were statistically significant compared with the negative control group, as presented in Table 10.

#### 3.9.7 Histopathological Examination

The histopathological examination of vital organs, including the heart, liver, and kidneys, following treatment with different doses of MSE (250, 500, and 1000 mg/kg) for 28 days revealed no significant alterations in the normal physiological structure compared to the negative control group. As shown in Figure 6, the examination of heart sections (Figure 7A–D) indicated that all doses of MSE preserved the normal morphological structure without signs of necrotic debris, interstitial edema, inflammation, or fibrosis. Similarly, liver sections (Figure 7E–H) displayed intact architecture and no pathological changes. The kidney sections (Figure 7I–L) also showed normal histological features with no evidence of damage or dysfunction. These findings suggest that MSE does not adversely affect the histological integrity of these vital organs at the administered doses.

RETRACTED

**FIGURE 7:** Photomicrograph presenting histopathology of the heart (A–D), liver (E–H), and kidney (I–L) at 10× of mice after the administration of MSE.

## 4 Discussion

The nutritional analysis of mango seed extract (MSE) revealed a notable nutritional profile, with significant levels of crude protein (8.5% ± 0.01%), crude oil (13.5% ± 0.06%) and fiber (2.8% ± 0.02%), carbohydrate (35% ± 0.01%), ash (1.8% ± 0.05%), and 405 kJ/100 g. The high carbohydrate content suggests that MSE could serve as a potential source of energy, while the presence of crude protein contributes to its nutritional value, potentially providing essential amino acids. The crude oil content is also noteworthy, as mango seed oil has been reported to contain beneficial fatty acids, making it a potential alternative to conventional vegetable oils.

The mineral content of MSE, including calcium, magnesium, potassium, sodium, and phosphorus, further enhances its nutritional significance. These minerals play crucial roles in various physiological processes, such as bone health (calcium and phosphorus), muscle function (potassium and magnesium), and electrolyte balance (sodium and potassium). The presence of these minerals suggests that MSE could be a valuable source of micronutrients, particularly in regions where dietary deficiencies are prevalent (Kemegne et al. 2018). Calcium contributes to teeth growth, regulating heartbeat, nerve impulse conduction, stimulating hormonal secretions, blood coagulation, and maintaining bone health (Townsend et al. 2011). In the same way, magnesium is a vital mineral for enzyme action and also aids in the management of many diseases, such as hypertension, acute heart attacks, chronic heart disease, arrhythmias, diabetes, asthma, chronic fatigue syndrome, and preeclampsia and eclampsia of pregnancy as calcium and chloride (Townsend et al. 2011). Phosphorus is required for the maintenance of the body's acid–alkaline balance, kidney function, and cell and bone development (Swaroop et al. 2018). Vitamins enhance the antioxidants' ability. Vitamin A is essential for normal vision, gene expression, growth, and immune function through its conservation of epithelial cell function. Vitamin C acts as a powerful antioxidant that enables the transference and uptake of nonheme iron at the mucosa, in the reduction of folic acid intermediates and cortisol synthesis (Kalupahana et al. 2018). Vitamin E acts as a powerful antioxidant that aids in protecting cells from injury by free radicals, and it is important for the formation and normal functioning of red blood cells and muscles. Vitamin K is an important factor in the regulation of blood coagulation; it causes slow tumor growth and inhibition of arterial calcification and stiffening (Sferrazzo et al. 2022). Therefore, the mango seed can be used as an unconventional source of vitamins and minerals. The qualitative phytochemical examination showed the occurrence of alkaloids, flavonoids, tannins, and triterpene, while steroids, saponins, and phalobatannins were absent. This approach provided a foundational understanding of the phytochemical profile of MSE and helped in subsequent biological evaluations. In another study, the quantitative evaluation by HPLC was done for the estimation of phytochemicals present in MSE (Saleem et al. 2023), while the current work was planned to extend this by estimating the antioxidant and in silico interactions of these bioactive compounds.

RETRACTED

In the case of the bio‐organic molecule, the functional group imparts specific biological activities that are responsible for its characteristics, such as acid–base properties, solubility, crystal configuration, partition coefficient, and stereochemistry. Hypothetically, all these characteristics are responsible for absorption, distribution, metabolism, excretion, and toxicity and for the prediction of structure–activity relationships of the bio‐organic molecule [48]. In the present study, the FTIR spectral evaluation of mango seeds revealed the existence of phytochemicals possessing a hydrogen‐bonded –OH functional group. It is well recognized that the –OH functional group is an important part of many phenolic compounds, for instance, flavonoids and tannins that impart antioxidant properties in the extract (Jung et al. 2024). Our inference showed that the given extract possesses numerous biologically active functional moieties such as alcohol, ester, aldehyde, and nitro compounds that confirm the presence of bioactive phytochemicals.

The most established, practical, and sensitive in vitro method for appraisal of the antioxidant potential of a given plant extract is based on the generation of the radical chromophore that excites the reactive oxygen species and purple‐colored free radical of DPPH (Itoh et al. 2020). The results of MSE at a concentration of 100 μg/mL showed a better free radical scavenging activity (95.86% ± 2.31%) followed by ascorbic acid (92.55% ± 4.70%). This inference of the present study is comparable to the investigational research conducted on the evaluation of the antioxidant character of mango kernel (Abdel‐Aty et al. 2018). The interspecies difference might be responsible for this variation. Nitric oxide (NO) acts as an important diffusible free radical produced by numerous cells, such as endothelial cells, macrophages, and neurons. It is responsible for numerous biological activities as an effector molecule. The reactive nitrogen species produced a reaction with oxygen or superoxides (NO_2_, N_2_O_4_, N_3_O_4_, NO_3_) are accountable for changes in the structural and functional activities of numerous cellular components (Sferrazzo et al. 2022). The nitric oxide scavenging activity in the present study was 80.45%, which is slightly less than ascorbic acid (89.36%) and imparts antioxidant potential to MSE.

RETRACTED

Phytotherapy is used for the treatment of different diseases (Sun‐Waterhouse et al. 2024). It is gaining encouragement due to strategies designed for its rational utilization and evaluation of the safety profile. The toxic potential and extent of adverse reactions were presented through the results of the toxicant and cell interaction. The toxicity profile is characterized to fulfill the requirements of regulatory agencies such as the WHO and the FDA by repeated exposure to substances (Buhari and Muhammad 2022). Although MSE possesses valuable pharmacological properties, it is deficient in comprehensive knowledge regarding the evaluation of subacute toxicological studies. In the current study, after subacute toxicity treatment, all experimental animals remained alive, active, with normal behavior according to the species, responsive toward stimuli, and had normal consumption of food and water intake, and no sign of clinical toxicity was seen in contrast with the negative control group. The toxic influence of the administered drug was shown by the vital organs through the existence and extent of clinical observation and symptoms. The organ damage manifested as an alteration in the organ‐to‐body weight ratio. The increase in vital organ weight has been associated with the toxicity of hepatic or nephrotic tissues. The outcome of the current investigation revealed no harmful effect on the weight of the liver, kidney, and heart. Evaluating the performance of the liver and kidneys presents a vital index in the assessment of the toxicity of plant extracts. It is evaluated through certain indicators of the liver (ALT, AST, bilirubin total, alkaline phosphatase, globulin, total protein, and albumin) and kidney (serum creatinine and urea) (Hussein et al. 2021). The consequences of the current investigation showed a statistically nonsignificant alteration in biomarkers of the liver and kidney in contrast to the negative control group. The data of the current investigation align with the findings of Yang et al. (2019).

Extract produces a statistically significant rise in HDL and a fall in LDL value in all treatment groups compared to vehicle control, which gives a clue to its cardioprotective property. Increased values of cholesterol, LDL, and VLDL are associated with tissue damage caused by tumors or any other disease. The present results align with the reported data that the hypolipidemic potential of the leaf extract of *Pachyptera hymenaea* in rats; the extract elevated the HDL levels and produced a decline in LDL levels (Arshad et al. 2021). Hematological parameters are susceptible biomarkers of any physiological alteration by toxicants in animals. The hematopoietic parameters of the current study present no toxic inference. The increase in RBC and Hb value suggests that the extract has a slight hemopoietic potential by increasing the physiological transportation of oxygen and carbon dioxide, possibly through improvement in erythropoiesis or reduction in RBC destruction. The phytoconstituents of the MSE exhibit the occurrence of alkaloids, flavonoids, and phenols that may be involved in the production of blood and can be used for the management of anemia (Torres‐León et al. 2016; Abdel‐Aleem et al. 2019). The exact mechanism behind this property is still uncovered. A statistically significant rise in WBC and lymphocyte counts at doses of 500 and 1000 mg/kg suggested an improvement in the activity of the immune system; therefore, its administration may decrease the risk of infection. Consequently, the observed increment in WBC count revealed possible augmentation of the leukopoietic and immunomodulatory properties of the extract. The current results align with the outcome of hematopoietic results and the antianemic potential of the leaf extract of *Hedranthera barteri* in rats (Karrat et al. 2022). Histopathological examination revealed no pathological alteration on a macro and microscopic scale in organs of animals receiving MSE at all doses 250, 500, and 100 mg/kg, respectively. No significant alteration was seen in the architecture of vital organs like the heart, liver, and kidney compared with the vehicle control group. These findings are supported by a research study that presented acute and subacute toxicity of the ethanolic extract from aerial parts of *Epigynum auritum* in mice (Karrat et al. 2022).

RETRACTED

The IC_50_ value of the MSE was 140 μg/mL. Various phenolic and polyphenolic components from the MSE have been reported to be efficient cytotoxic agents. These include naringenin, verbascoside (acetoside), chgenin, and kaempferol 3‐O‐glucoside (Kumar et al. 2021). Several research works have pointed out that mango seed kernel has been recognized as a good source of natural antioxidants (Abdalla et al. 2007; Jahurul et al. 2015).

Our findings are consistent with earlier research that demonstrated the ability of MSE extracts to stop the growth of human cancer cells (Mahmoud et al. 2024). The data obtained from the GC–MS analysis of MSE revealed the existence of different compounds. While GC–MS is a widely used technique for the identification of volatile and semi‐volatile phytochemicals, it is characteristically limited in its ability to detect nonvolatile, thermolabile, or high‐molecular‐weight compounds, such as glycosides, tannins, and certain flavonoids. These compounds either degrade at high injector temperatures or are not efficiently volatilized, thus escaping detection by GC–MS (Sasidharan et al. 2011; Pandey and Tripathi 2014). As a result, the GC–MS profile of MSE may not reflect the full spectrum of bioactive constituents, particularly those with higher polarity or thermal instability. All these identified constituents revealed their biological actions, such as anticancer, antiandrogenic, and anticoronary potential. Some of these bioactivities reported in the literature were directly related to antiproliferative properties, protection against oxidative stress, and anti‐inflammatory potential. The results are comparable to those of the previous studies that showed the existence of various phytochemicals in MSE (León‐Roque et al. 2023).

To explore the potential therapeutic relevance of bioactive compounds identified in MSE, molecular docking and MDS were conducted. Selected phytochemicals‐[thiazole, 2‐ethylacridine, silicic acid, 3,5‐ethanoquinolin‐10‐one, hexahydropyridine] were chosen based on their prevalence in the extract and suspected biological activities. These ligands were docked against protein targets [Estrogen_receptor_beta_9256; Progesteron_9256] which are implicated in inflammation or oxidative stress—conditions that cause breast cancer, endometrial cancer, and neurological diseases. The stability of the complex was demonstrated by the time‐dependent fluctuation in root mean square deviation (RMSD) values for C‐alpha atoms in ligand‐bound proteins. Differences in ligand RMSD over time are plotted along the right *Y*‐axis. Protein RMSD shifts over time are plotted on the left Y‐axis. According to the RMSD, from the start, the complex shows some stability. From 20 ns, the compound shows some fluctuations and increases slightly. Conversely, from 10 ns, the RMSD of the protein‐bound ligand shows stability. No significant variation or modification was seen after 10 ns in the simulated protein–ligand fit analyses. The RMSD displayed fluctuations, but the ligand, after equilibrium RMSD computation, did not reveal any significant alterations. This showed the stability of the receptor and compound complex. The root mean square fluctuation (RMSF) value of the protein–ligand complex was calculated. During the simulation, the secondary structure elements, such as beta‐strands and alpha‐helices, were anticipated. The ratio of beta‐sheets and alpha‐helices also influences the protein's RMSD. The RMSD of the residues in these structures was lower than that of the residues located in coils and loops because the protein contains rigid regions. Most of the significant ligand–protein interactions were made up of hydrogen bonds. The interaction between the target protein and the chosen ligand was revealed by the molecular contacts and interactions (H bonds, hydrophobic, ionic, and water bridges). In Figure 6G, hydrogen bonding was observed for GLU_305 residues. Hydrophobic bonding was observed for PRO_277, TRP_312, and TRP_345 residues. Hydrophobic bonding was also observed for LEU_715 and PHE_905 residues. The ligand–protein interaction was also critically observed throughout the simulation analyses.

RETRACTED

## 5 Conclusion and Future Prospects

This study demonstrates that mango seed extract (MSE) is a rich source of bioactive compounds, including essential amino acids, vitamins, and antioxidants, which collectively contribute to its potent nutraceutical properties. The extract exhibited significant antioxidant activity and cytotoxic effects against HepG2 liver cancer cells, highlighting its potential as a natural therapeutic agent. Importantly, subacute toxicity assessments confirmed the safety of MSE at doses up to 1000 mg/kg, with no adverse effects observed on vital organ weights, histopathology, or hematological parameters. Additionally, MSE positively influenced lipid profiles by reducing harmful cholesterol fractions and enhancing beneficial HDL levels, suggesting cardiovascular benefits.

Looking forward, these promising findings warrant further investigation to fully elucidate the molecular mechanisms underlying MSE's bioactivities. Future studies should focus on isolating and characterizing individual bioactive constituents to determine their specific roles and synergistic effects. Moreover, in vivo efficacy trials in relevant disease models, including cancer and metabolic disorders, are essential to validate therapeutic potential and optimal dosing strategies. Long‐term toxicity and pharmacokinetic studies will also be critical to ensure safety and bioavailability in humans.

From an industrial perspective, the valorization of mango seed waste into high‐value nutraceutical products offers an eco‐friendly and sustainable approach to reduce agricultural by‐products. Developing standardized extraction methods and formulation strategies will facilitate the incorporation of MSE into functional foods, dietary supplements, and pharmaceutical applications. Ultimately, this research lays a strong foundation for translating mango seed extract into practical health‐promoting interventions, contributing to both human well‐being and environmental sustainability.

RETRACTED

## Author Contributions

S.I. performed the methods and investigation. E.Z., I.A.M.A., and R.C.‐M. conceptualized and funded the acquisition, whereas M.U.R. and H.R. supported the original drafting of the manuscript. Z.S. and M.F. wrote the original draft and provided supervision in the analysis. M.A.R., H.A.Z., and R.C.‐M. wrote the review and editing, R.A., S.G., A.K., and Y.B. provided visualization. All authors have read and agreed to the published version of the manuscript.

## Disclosure

Declaration: I hereby declare that this research work has not been published elsewhere, nor is it under consideration for any other publication.

## Conflicts of Interest

The authors declare no conflicts of interest.

## Data Availability

Data are contained within the article.
